The article "Evaluation of Pericapsular Nerve Group (PENG) Block for Analgesic Effect in Elderly Patients with Femoral Neck Fracture Undergoing Hip Arthroplasty" was retracted in 2023. Reasons: signs of a paper mill; suspected computer-generated content; unreliable results or conclusions; concerns about the data.

# Evaluation of Pericapsular Nerve Group (PENG) Block for Analgesic Effect in Elderly Patients with Femoral Neck Fracture Undergoing Hip Arthroplasty

**DOI:** 10.1155/2022/7452716

**Published:** 2022-02-09

**Authors:** Hao Hua, Yan Xu, MengLu Jiang, Xu Dai

**Affiliations:** Department of Anesthesiology, Wuxi Ninth People's Hospital, Wuxi 214062, China

## Abstract

**Background:**

For evaluating pericapsular nerve group (PENG) block's analgesic effect on elderly patients suffering from femoral neck fracture undergoing hip arthroplasty to provide a basis for optimizing perioperative analgesia in hip arthroplasty.

**Methods:**

Forty-eight patients undergoing hip arthroplasty with spinal anesthesia for femoral neck fracture in our hospital were chosen in this study. Based on the random number table method, patients were categorized into the following two groups (*n* = 24 per group): the hip peripheral nerve group block group (PE group) and the iliac fascia block group (FI group). The fascia iliaca compartment block was used in the FI group, whereas the pericapsular nerve group block in the PE group. When placed in the position for spinal anesthesia (T4), we measured dynamic and static visual analog scale (VAS) scores as well as analgesic satisfaction before blockade (T0), along with at 10 min (T1), 20 min (T2), and 30 min postblockade (T3). Sufentanil dosage and effective analgesic pump press number at 6 h (T5), 12 h (T6), 24 h (T7), and 48 h (T8) postoperatively were recorded. In the meantime, the development of related complications was also recorded.

**Results:**

Compared with T0, patients in both groups achieved lower static VAS scores at T1–T4 (*P* < 0.05) and lower dynamic VAS scores at T2–T4 of the FI group (*P* < 0.05). Relative to the FI group, both static and dynamic VAS scores at T1–T4 were obviously lower in the PE group (*P* < 0.05), along with increased dynamic analgesic satisfaction (*P* < 0.05). Weakness of the quadriceps was observed in seven patients in the FI groups (*P* < 0.05). No delirium, hematoma, puncture site infection, or nerve injury occurred in either group.

**Conclusion:**

The pericapsular nerve group block can provide safe and effective analgesia for elderly patients during the perioperative period of hip arthroplasty, with rapid onset, good analgesic effect, high patient satisfaction, and low complication rate, and is worthy of widespread application. The trial is registered with ChiCTR2100046785.

## 1. Background

Hip arthroplasty is the main surgical treatment for femoral neck fractures in the elderly, and given China's aging population, hip arthroplasty is frequently performed in clinical practice. [1, 2] Numerous studies have shown that hip arthroplasty can cause severe pain in the perioperative period, which can lead to a series of related complications, which not only increases the perioperative risk but also is detrimental to the long-term prognosis of patients. Therefore, an optimal perioperative analgesia can greatly facilitate the patient's postoperative recovery. [3, 4] The fascia iliaca compartment block is often used to relieve patients' perioperative pain; however, numerous studies and prior clinical work have identified the risks of neurovascular injury, quadriceps weakness, and delayed recovery. [5, 6] The sensory nerve pattern of the hip capsule is different in anterior or posterior regions. The anterior hip capsule contains most sensory fibers and mechanoreceptors. [7] The anterior capsule of the hip has been innervated by the femoral nerve (FN) and the foramen ovale (ON) branches. The articular branch of the FN provides most of the innervation to the lateral and superomedial aspects of the hip capsule, whereas the branch of the ON innervates the medial portion of the capsule. The proximal articular branches of the FN and ON locate all the way between iliopubic eminence and anterior inferior iliac spine, while the ON is located close to medial acetabulum, near the medial aspect of the acetabulum. The posterior hip capsule surface is innervated with sciatic nerve branch: superior gluteal nerve and the nerve of the quadriceps muscle. [8, 9] The pericapsular nerve group (PENG) block refers to a new regional block technology providing analgesia by blocking branches from FN, ON, and accessory obturator (AON). [10] It should only target the anterior branch to the hip joint. Sensory branches from FN appearing distal to the groin are reasonably excluded from this block. Therefore, it can achieve the ideal analgesia without affecting the patient's muscle strength, thus facilitating the patient's postoperative functional recovery. [11] A distinct advantage of the PENG block is the supine position, which is especially important for patients with chronic pain or acute hip fractures. However, these studies are mostly case reports. The current work compared the analgesic effect and safety of fascia iliaca compartment block (FICB) and PENG block in elderly patients undergoing femoral neck fractures during the perioperative period and provided a reference for clinical application.

The article "Evaluation of Pericapsular Nerve Group (PENG) Block for Analgesic Effect in Elderly Patients with Femoral Neck Fracture Undergoing Hip Arthroplasty" was retracted in 2023. Reasons: signs of a paper mill; suspected computer-generated content; unreliable results or conclusions; concerns about the data.

## 2. Materials and Methods

This study got approval from the Ethics Committee of Wuxi Ninth People's Hospital (ID: LW2021012) and registered on 28 May 2021 (retrospectively registered) on the Chinese Clinical Trial Registry (ID: ChiCTR2100046785). This work was a single-center, single-blind, prospective, randomized controlled trial. A total of 48 (27, male; 21, female) patients with the age of 65–85 years, the body mass index (BMI) of 20–30 kg/m^2^, and with the American Society of Anesthesiologists (ASA) physical status II–III undergoing hip arthroplasty due to femoral neck fracture in our hospital from April 2020 to April 2021 were selected. Moreover, 26 and 22 patients underwent hemi hip arthroplasty and total hip arthroplasty, respectively. Besides, a random number table was applied to category groups in the pericapsular nerve group block group (PE group) and the fascia iliaca compartment block group (FI group), with 24 patients in each group. All patients provided written informed consent.

### 2.1. Exclusion Criteria

The following presents the exclusion criteria: people with ① a history of mental or neurological disorders that prevent normal communication, ② coagulation disorders, ③ serious cardiovascular diseases,④ mental illness or hearing impairment and aphasia and who were unable to communicate, ⑤ puncture site infection, ⑥ a history of allergy to local anesthetic drugs, ⑦ neuromuscular lesions of the lower extremities, and ⑧ a history of epilepsy and alcoholism.

### 2.2. Randomization and Blinding

A nurse not involved in the study used a computerized random number generator to generate random numbers for either the PE or PI group at the ratio of 1 : 1. The randomization sequence was placed in sealed opaque envelopes, and the trial operation was blocked by an experienced anesthesiologist. Group assignment was confidential to the investigator who assessed the quality of the block. A resident anesthesiologist who was confidential to the randomization assignment shoulder the responsibility for gathering intraoperative data. Another investigator, namely, independent of group assignment, was responsible for collecting postoperative data. In the end, a statistician carried out the statistical analysis and kept the entire process confidential [12].

### 2.3. Anesthesia Method

Patients were admitted to the operating room with routine cardiac monitoring and open intravenous access. Patients in both groups were located in the supine position, and ultrasound-guided puncture was performed by the same experienced anesthesiologist. Methods of operation in the PE group were as follows: patients were operated with a curvilinear low-frequency ultrasound probe (SonoSite Edge II, frequency: 2–5 MHz) placed vertically within transverse plane where anterior inferior iliac spine is located. Subsequently, the probe was rotated counterclockwise approximately 45° to align with the pubic ramus. The iliopsoas tendon, iliopubic eminence, femoral artery, iliopsoas muscle, and pectineus muscle can be observed in this plane. By employing an in-plane approach, a 22-gauge 80-mm nerve stimulation needle was inserted from outside to inside, and the tip was placed on myofascial plane between posterior pubic ramus and anterior iliopsoas tendon (Figure 1), and 0.4% ropivacaine 20 mL was injected after backdrawing without blood. The methods of operation in the FI group were as follows: patients assumed the supine position and were operated using the high-frequency ultrasound probe (SonoSite Edge II, frequency: 5–13 MHz), which was positioned at the inguinal ligament vertical to the ligament. A short needle was used to penetrate the fascia lata and iliac fascia to reach iliac fascia. After the extraction of no blood, 4 mL of normal saline was inserted. After the correct position was verified, 30 mL of 0.4% ropivacaine hydrochloride was inserted. After the nerve block, both groups of patients received spinal anesthesia injection. Patients were turned to the lateral position with the affected side underneath, routinely disinfected with towels, and infiltrated with 2% lidocaine local anesthesia, with the L3∼L4 space used as the puncture site. Moreover, 2–2.5 mL of 0.5% bupivacaine hydrochloride was injected after puncture, and cerebrospinal fluid flow was observed, after which the patient was placed supine and the procedure was started. After surgery, patient-controlled intravenous analgesia was infused, with the following drug configurations: sufentanil 100 *μ*g + tropisetron 10 mg, diluted to 100 mL with saline, with a background dose of 1 mL/h, a self-controlled dose of 2 mL each time, lock time of 15 min, and use time of 48 h. If the patient's analgesic requirements are not met while the drug is administered according to the study protocol during the observation period, the patient may request remedial analgesia, intravenous oxycodone 1 mg.

The article "Evaluation of Pericapsular Nerve Group (PENG) Block for Analgesic Effect in Elderly Patients with Femoral Neck Fracture Undergoing Hip Arthroplasty" was retracted in 2023. Reasons: signs of a paper mill; suspected computer-generated content; unreliable results or conclusions; concerns about the data.

### 2.4. Observation Indicators

All data collection and processing were performed by another anesthesiologist who was not involved in the infusion of anesthesia. (a) Visual analog scale (VAS) scores were adopted for evaluating patients' level of pain (0, no pain; 10, severe pain). The patients' static VAS scores before the nerve block (T0) and static and dynamic VAS scores (passive leg raising 15°) at 10 min (T1), 20 min (T2), and 30 min (T3) after the nerve block and before the start of spinal anesthesia infusion (T4) were recorded. (b) Patient satisfaction scores (4, very satisfied; 3, satisfied; 2, fair; and 1, unsatisfied) for analgesia were recorded at the end of the operation. The cumulative dosage of sufentanil and the effective number of analgesic pump presses at 6 h (T5), 12 h (T6), 24 h (T7), and 48 h (T8) postoperatively were recorded, and the occurrence of adverse reactions such as delirium, hematoma, puncture site infection, nerve injury, rescue analgesics situation, and Quadriceps strength during analgesia was observed. Quadriceps muscle strength testing method is described as follows: the patient is in supine position; the examiner supports the knee joint with one hand under the popliteal fossa; the other hand exerts resistance on the patient's lower leg and asks the patient to extend the knee joint to resist the resistance; if the knee joint cannot be extended, it means that the quadriceps muscle is weak; first, the surgical side of the limb is measured, and then, the nonsurgical side of the limb is measured.

### 2.5. Data Analysis

The sample size was measured according to our preliminary study of totally 20 patients (10 in each group). Our preliminary study showed a cumulative VAS score at 30 minutes postanesthesia of 3.2 ± 0.4 in the FI group and 2.9 ± 0.3 in the PE group. The sample size was 21 in each group (*α* = 0.05, power = 0.8). Given a follow-up loss rate of nearly 10%, this study registered 24 subjects in each group (Figure 2).

All statistical data analyses were performed with the application of SPSS software, version 25.0 (SPSS Inc, Chicago, IL, USA). Normally distributed measures are denoted as mean ± standard deviation ($\bar{x}+s$). The *T*-test was applied to make independent comparisons between groups. In the meanwhile, the paired *t*-test was employed to perform intragroup comparisons. Moreover, the *χ*^2^ test was applied for making the comparison of count data. The differences were regarded to present statistical significance at *P* < 0.05.

## 3. Results

There existed no statistically obvious difference between the two groups regarding general conditions such as age, sex ratio, BMI, operation time, and ASA classification (*P* > 0.05, Table 1).

In comparison with T0, patients in both groups had lower static VAS scores at T1–T4 (*P* < 0.05) and lower dynamic VAS scores at T2–T4 in the FI group (*P* < 0.05) and lower dynamic VAS scores at T1–T4 in the PE group (*P* < 0.05). In comparison with the FI group, static and dynamic VAS scores at T1–T4 were lower (*P* < 0.05) and analgesic satisfaction scores remained higher (*P* < 0.05, Figures 3–5) in the PE group.

There existed no statistically obvious difference between the cumulative sufentanil dosage and the number of analgesic pump presses at T5–T8 in the two groups (*P* > 0.05, Table 2). No significant difference in VAS scores after surgery ((*P* > 0.05, Figure 6).

Weakness of the quadriceps was observed in seven patients in the FI group (*P* < 0.05, Table 3).

The article "Evaluation of Pericapsular Nerve Group (PENG) Block for Analgesic Effect in Elderly Patients with Femoral Neck Fracture Undergoing Hip Arthroplasty" was retracted in 2023. Reasons: signs of a paper mill; suspected computer-generated content; unreliable results or conclusions; concerns about the data.

## 4. Discussion

Spinal anesthesia is preferred as the anesthetic method for hip arthroplasty in elderly patients, and the commonly used analgesic method is FICB, which is easier to operate and has better analgesic effect than intravenous fentanyl and nonsteroidal analgesics alone. [13] However, in clinical practice, there is an insufficient analgesic effect is observed after the application of FICB. Some studies [14] have observed the diffusion of local anesthesia using FICB under magnetic resonance imaging and showed that the diffusion of local anesthesia using FICB did not successfully block the obturator. This indicates that FICB could not completely relieve the hip pain. The anterior hip capsule is mainly innervated by sensory fibers originating from the FN, ON, and AON and is a key target for hip analgesia. [15] The PENG block is based on the anatomical study of the hip nerve and identifies a regional analgesic method that uses the nerve associated with the anterior hip capsule as a key target, providing rapid and effective relief of hip pain without increasing adverse effects [10].

The results of this study showed that both static and dynamic VAS scores at T1–T4 tended to decrease in both groups within 30 min of the implementation of the two analgesic methods, indicating that both blocking methods were effective in relieving acute early pain in elderly patients suffering from hip fracture. Compared with T0, the static and dynamic VAS scores were lower in the PE group from T1 to T4. In addition, the dynamic VAS scores were lower in the FI group from T2 to T4. Moreover, the static and dynamic VAS scores were obviously lower in the PE group in comparison with the FI group at 10 min after the block, implying that the PENG block had a faster onset of action compared with the FICB. The static and dynamic VAS scores of the PE group were lower compared with those in the FI group at T1–T3, which demonstrated that the analgesic effect of PENG block was better than FICB. In comparison with the FI group, the PE group had lower static and dynamic VAS scores and higher dynamic analgesic satisfaction at T4, probably because the PENG block was better for the closed nerve compared with the FICB. Usually, patients with femoral neck fractures have difficulty in body position placement prior to spine anesthesia due to severe pain in the hip, and the success rate of anesthesia operations is subsequently reduced. Moreover, the severely painful movement caused by the body position placement increases the patient's stress response and tends to cause fluctuations in circulatory function, thus increasing the risk of anesthesia. In this study, VAS scores were obviously lower in the PE group compared with those in the FI group after the block was performed, indicating that the PENG block was more effective in analgesia. Moreover, it facilitated the positioning of the patient before anesthesia, thus improving the comfort of the patient with spinal anesthesia. This indicates that PENG block can provide more convenient conditions for the smooth implementation of spinal anesthesia.

The article "Evaluation of Pericapsular Nerve Group (PENG) Block for Analgesic Effect in Elderly Patients with Femoral Neck Fracture Undergoing Hip Arthroplasty" was retracted in 2023. Reasons: signs of a paper mill; suspected computer-generated content; unreliable results or conclusions; concerns about the data.

In addition to the FN, ON, and AON, the hip joint is similarly innervated by the articular branches of the sciatic and superior gluteal nerves. [16] Since both nerve block methods were unable to block the sciatic and superior gluteal nerves, a self-contained intravenous analgesic pump was used in both groups to assist in analgesia after surgery. According to the results, there existed no difference in the cumulative amount of sufentanil and the number of effective analgesic pump presses between the two groups, suggesting that pericapsular nerve group block can provide good postoperative analgesia. Moreover, the postoperative analgesic effect was similar to FICB. In this study, no patient in either group had adverse reactions such as puncture site infection and hematoma, suggesting that the application of the PENG block of the hip is safer than FICB. However, considering that the PENG block site of the hip joint is close to the hip joint, the principle of asepsis should be strictly observed during operation to prevent hip joint infection.

There is a direct relationship between postoperative pain and patient length of stay, with higher levels of pain associated with longer hospital stays. [17] Early removal from bed is more conducive to faster postoperative recovery and early discharge. [18] In this study, patients were assessed for quadriceps weakness by referring to the literature [19]. The results showed that the incidence of quadriceps muscle weakness was reduced in the PE group at 48 h postoperatively compared with the FI group. It is suggested that compared with FICB, the PENG block for total hip arthroplasty under spinal anesthesia in elderly patients does not affect postoperative quadriceps muscle strength and facilitates early postoperative recovery. Tran et al. [20] injected two volumes of methylene blue in 10 ml and 20 ml using the PENG block on cadaveric specimens. The results show although the diffusion pattern was more extensive with the 20 ml injection, both the 10 ml and 20 ml injections diffused within the interstitial space of the defined bursal between the iliopsoas and anterior hip joint capsule. Ahiskalioglu et al. [21] reported an ultrasound-guided PENG block with 30 ml of local anesthetic (0.5% bupivacaine 15 ml + 2% lidocaine 15 ml), demonstrating that the femoral nerve, obturator, and lateral femoral cutaneous nerve were blocked. The exact cause of this is unknown and needs to be further investigated. Meanwhile, the appropriate volume of local anesthetic still needs further study.

The article "Evaluation of Pericapsular Nerve Group (PENG) Block for Analgesic Effect in Elderly Patients with Femoral Neck Fracture Undergoing Hip Arthroplasty" was retracted in 2023. Reasons: signs of a paper mill; suspected computer-generated content; unreliable results or conclusions; concerns about the data.

One aspect that needs to be discussed is that although anterior capsule innervation is the cause of most hip-related pain, the PENG block provides analgesia only to the anterior capsule of the hip but neglects the posterior capsule. The posterior capsule is innervated by the nerve of the quadriceps and superior gluteal nerves emanating from the sacral plexus, which also have an important function in the complete analgesia of the hip capsule. Therefore, as some recent studies have pointed out [22], in future studies, we will use the PENG block compared with sciatic nerve blocks or other analgesic techniques as a way to provide complete analgesia of the hip capsule.

## 5. Conclusion

To summarize, from this study, it can be concluded that the pericapsular nerve group block is fast-acting, with a good analgesic effect and high patient satisfaction and can provide effective and good perioperative analgesia for elderly patients undergoing hip arthroplasty, which is worthy of widespread application.

## Figures and Tables

**Figure 1:** An ultrasound image of the PENG block (white arrow). AIIS: anterior inferior iliac spine, FA: femoral artery, IPE: iliopubic eminence, and PE: pectineus muscle.

**Figure 2:** Consolidated Standards of Reporting Trials (CONSORT) flow diagram.

**Figure 3:** Trends in static (a) and dynamic (b) VAS scores of the two groups. Note: *P* < 0.05 compared with the PE group, label^∗^; *P* < 0.05 compared with T0, label #; VAS, visual analog scale; PE, pericapsular nerve group block group; FI, fascia iliaca compartment block group.

**Figure 4:** Static and dynamic VAS scores at T4 of the two groups. VAS, visual analog scale; PE, pericapsular nerve group block group; FI, fascia iliaca compartment block group. Note: *P* < 0.05 compared with T0, label #.

**Figure 5:** Static and dynamic satisfaction of the two groups. PE, pericapsular nerve group block group; FI, fascia iliaca compartment block group.

**Figure 6:** Trends in static (a) and dynamic (b) VAS scores of the two groups after surgery. PE, pericapsular nerve group block group; FI, fascia iliaca compartment block group.

**Table 1:** Comparison of general information between the two groups ($\bar{x}\pm s$).

Group	Male/female	Age (years)	ASA classification (II/III)	BMI (kg/m^2^)	Surgery time (min)
PE group	14/10	74 ± 7	6/18	24 ± 3	133 ± 13
FI group	13/11	74 ± 8	7/17	23 ± 4	129 ± 19

ASA, American Society of Anesthesiologists; BMI, body mass index; PE, pericapsular nerve group block; FI, fascia iliaca compartment block.

The article "Evaluation of Pericapsular Nerve Group (PENG) Block for Analgesic Effect in Elderly Patients with Femoral Neck Fracture Undergoing Hip Arthroplasty" was retracted in 2023. Reasons: signs of a paper mill; suspected computer-generated content; unreliable results or conclusions; concerns about the data.

**Table 2:** Comparison of cumulative postoperative sufentanil dosage and effective number of analgesic pump compressions between the two groups ($\bar{x}\pm s$).

Group	Index	T5	T6	T7	T8
PE group	Sufentanil cumulative dosage (ug)	7.5 ± 1.0	18.5 ± 2.3	32.4 ± 5.8	82.3 ± 8.7
FI group		8.0 ± 1.2	19.3 ± 3.1	34.7 ± 4.1	85.4 ± 8.2
*t*		1.568	1.015	1.586	1.270
*P*		0.124	0.315	0.120	0.210
PE group	Number of effective compressions with analgesic pump	1.3 ± 0.7	2.7 ± 1.1	4.7 ± 1.7	10.8 ± 2.4
FI group		1.6 ± 0.6	3.2 ± 1.6	5.4 ± 1.9	11.4 ± 2.5
*t*		1.594	1.262	1.345	0,848
*P*		0.118	0.213	0.185	0.401

PE, pericapsular nerve group block; FI, fascia iliaca compartment block;

**Table 3:** Comparison of postoperative adverse reactions between the two groups.

Group	Delirium	Bloody swelling	Puncture site infection	Nerve injury	Quadriceps weakness	Rescue analgesics
PE group	0	0	0	0	0^*∗*^	0
FI group	0	0	0	0	7	0

Note: compared with the FI group, ^*∗*^*P* < 0.05. PE, pericapsular nerve group block; FI, fascia iliaca compartment block.

## Data Availability

The datasets generated and analyzed during the current study are available from the corresponding author on reasonable request.

## Abbreviations

ASA: American Society of Anesthesiologists
BMI: Body mass index
FI: Iliac fascia block
PE: Pericapsular hip nerve group block
VAS: Visual analog scale.

## Additional Points

*Trial Registration*. The study was registered on 28 May 2021 (retrospectively registered) on the Chinese Clinical Trial Registry: ChiCTR2100046785.
